The article "Queen cells acceptance rate and royal jelly production in worker honey bees of two Apis mellifera races" was retracted in 2022. Reasons: compromised peer review; a conflict of interest; concerns about the authorship.

# Queen cells acceptance rate and royal jelly production in worker honey bees of two *Apis mellifera* races

**DOI:** 10.1371/journal.pone.0248593

**Published:** 2021-04-13

**Authors:** Khalid Ali Khan, Hamed A. Ghramh, Zubair Ahmad, Mogbel A. A. El-Niweiri, Mohamed Elimam Ahamed Mohammed

**Affiliations:** 1 Research Center for Advanced Materials Science (RCAMS), King Khalid University, Abha, Saudi Arabia; 2 Unit of Bee Research and Honey Production, Faculty of Science, King Khalid University, Abha, Saudi Arabia; 3 Biology Department, Faculty of Science, King Khalid University, Abha, Saudi Arabia; 4 Biology Department, Faculty of Arts and Sciences, Zahran al-Janobe, King Khalid University, Abha, Saudi Arabia; 5 Department of Chemistry, Faculty of Science, King Khalid University, Abha, Saudi Arabia; Harran Üniversitesi: Harran Universitesi, TURKEY

## Abstract

Royal jelly (RJ) is an acidic yellowish-white secretion of worker honey bee glands, used as food material of worker bee larvae for the first three days and queen bee larvae for the entire life. It is commercially used in cosmetics and medicinal industry in various parts of the world. This study determined the queen cell acceptance rate and RJ production difference among Italian and Carniolan bee races. Furthermore, the effect of plastic cup cell priming media, diets and seasons were tested on the larval cell acceptance rate and RJ yield of both races. The results indicated that average queen cell acceptance rate was significantly (p<0.001) higher in Italian race (75.53 ± 1.41%) than Carniolan race (58.20 ± 1.30%). Similarly, mean RJ yield per colony significantly (p<0.001) differed between both bee races, which were 13.10 ± 0.42 g and 9.66 ± 0.43 g, in Italian and Carniolan races, respectively. Moreover, priming media, diets and seasons significantly (p<0.001) affected queen cell acceptance rate and RJ production of both bee races. This study would help breeders to select the bees with higher-level of queen cell acceptance rate and RJ production in the future.

## Introduction

Royal jelly (RJ) is a yellowish-white proteinaceous secretion of mandibular glands (MGs), hypopharyngeal glands (HGs), postcerebral, and thoracic glands of young nurse bees [1–4]. It is an acidic substance with pH of 3.4–4.5 and possesses a distinct sweet-sour taste with pungent smell [5]. The RJ is a nutritive substance for worker and drone larvae for the first three days and used as a food for queen bees throughout their larval stages [6]. The RJ contributes to unique qualities of queens such as longevity, high fertility, excellent learning and memory ability [7]. Furthermore, RJ has a unique source of precious natural ingredients with cosmetics potential activities and health-promoting properties [5, 8, 9]. The RJ is reported as a potential medicine used as anti-aging [10], anti-cancer [11], anti-diabetic [12], and improve postmenopausal pathologies [13] and cognitive ageing and Alzheimer’s disease [14].

The RJ can be produced on commercial basis as its market value is higher than other bee products, including honey, pollen and propolis. Nonetheless, RJ has become a major income source of beekeepers around the world [15–20]. For instance, China is one of the largest producers and exporter of RJ harvesting 4000 tons annually, accounting for >90% global RJ production. It is mostly exported to the USA, Europe, and Japan [21–23]. Some other countries and regions, including Vietnam, Taiwan, Korea and Japan are important producers and exporter of RJ. It is also produced in Eastern and Western Europe such as Greece, Spain, France and Italy as well as in Mexico [22, 24].

Various biotic and abiotic factors affect the quantity and quality of RJ [25–28]. The most important factors are honey bee races [23, 29], colony type, i.e., queen-less or queenright [30], transfer age of the larvae [31], number of transfer queen cell cup [30, 32], grafting techniques [33], grafting bar level and queen cell position [34, 35], harvesting interval [36], feeding source [37–39] and seasons [25, 35, 40]. For instance, when bees are fed on sugar syrup, it causes significant changes in the amount and structure of vital components of RJ such as amino acids, carbohydrates and vitamins [41]. The apiculture scientists are making significant efforts to develop different tools, grafting techniques to select high-producing strains of the honeybee for increasing RJ production.

The present study was conducted to compare the queen cell acceptance rate and RJ production difference between Italian and Carniolan bee races. Moreover, the effects of various priming media, diets and seasons on larval acceptance rate and RJ production between tested races were investigated. It was hypothesized that the tested bee races will significantly differ for the studied traits. The results will help in the selection of bee race with higher RJ production potential.

## Materials and methods

### Queen cell acceptance rate and royal jelly production

Five colonies per race with a standardized adult population size, food store and brood pattern were used to compare larval acceptance rate between Italian (*Apis mellifera ligustica*) and Carniolan (*A*. *mellifera carnica*) bee races. Queenright colonies were prepared by using queen excluder above the chamber confining the queen and rearranging the frames as in queenless builders. Six frames with uniform developmental stages and equal population of bees were placed in queen-less hive. The grafting frames were placed in the rearing colonies before grafting for polishing. Young worker larvae (<24 h old) were grafted into one frame containing 126 plastic queen cell cups fixed on two strips of wooden bars, which was introduced to the colonies of both races. After 3 days, the frame was taken out from the colony to check the queen cell acceptance and RJ production, according to standard procedures [42, 43]. The adult bees were removed from the frame and queen cell acceptance rate were determined by counting the proportion of queen cells containing the larvae and RJ.

The wax at the top of the plastic cells and larvae in the cells was removed. The RJ was collected from all cells with a micro spatula in a plastic container, and weighed on an electronic scale (AL204-IC, Mettler Toledo, Switzerland). The collected RJ was placed in the container and saved in refrigerator for future use. This experiment was repeated three times with three-day intervals.

### The impact of various priming media on larval acceptance rate and RJ production

Five different priming media were used to determine the queen cell acceptance and RJ production of tested bee races. Two colonies with standardized adult population size, food store and brood pattern were selected for each treatment. Firstly, queen plastic cell cups were treated with RJ alone, diluted RJ (1:1 with water), honey solution (1:1 with water), sugar syrup (1:1 with water), distilled water and dry (control). Afterwards, < 24 h-aged worker larvae were grafted into one frame containing 126 plastic queen cell cups fixed on two strips of wooden bars, which was introduced to both races. After 3 days, the frame was taken out from the colony to check the queen cell acceptance and RJ production, according to the standard procedures as described above [42, 43].

### The effect of various diets on queen cell acceptance rate and RJ production

To determine the effect of various diets on queen cell acceptance and RJ production, colonies were divided into equal groups that received following treatments. The first group was provided with pollen from a natural source, second group was fed on pollen substitutes (soybean flour + brewer’s yeast powder). Whereas, only sugar syrup was provided to bees as a control to third group. The artificial diets were placed on the brood frames in experimental bee colonies. Two colonies were used for each diet with three replications.

### The effect of seasons on larval acceptance rate and RJ production

Three colonies of each bee race were selected to determine the effect of seasons on queen cell acceptance rate and RJ production. The colonies were chosen with the same adult population size, food store and brood pattern. In each colony, the queen bee was removed 48 h before the grafting process. Queen cell acceptance rate and RJ production were calculated between both races during summer and winter season, according to standard procedures [42, 43].

### Statistical analysis

The data were analyzed by using SPSS software (version 26) and analysis of variance (ANOVA) was implied. Comparison between the races was performed by Student’s t-test to determine the significance. One-way ANOVA followed by Tukey post-hoc test was used to record difference between three or more groups. The data relating to queen cell acceptance rate means, RJ production means and other means were compared at 0.05 probability level.

## Results

### Queen cell acceptance rate

The difference of queen cell acceptance rate between both races was significant (Fig 1). The results revealed that the percentage of queen cell acceptance rate was significantly higher in Italian race as compared to Carniolan one (t = 9.016, p = 0.001). In contrast, there was no significant difference in queen cell acceptance rate within both bee races. The maximum queen cell acceptance rate was 75.53 ± 1.41% in Italian race, whereas the maximum queen cell acceptance rate was 58.20 ± 1.30% in Carniolan race.

**Fig 1:** Queen cell acceptance rate (shows as mean ± SE) of Italian and Carniolan bee races from 10 colonies (five colonies of each race) over three collection time points. “***” represents statistically significant differences (Student’s *t*-test, p<0.05).

### Royal jelly production

The mean weight of royal jelly per colony (g) and per cup (mg) between Italian and Carniolan bee colonies is given in Fig 2A and 2B. The RJ production was significantly higher in Italian race than Carniolan race (t = 5.765, p = 0.001). The highest RJ production was 13.10 ± 0.42 g in Italian race, whereas Carniolan race had 9.66 ± 0.43 g RJ production.

**Fig 2:** Mean weight (mean ± SE) of royal jelly for Italian and Carniolan lines around 72 hours after larval grafting (a) RJ production per colonies in grams after 72 h harvesting and (b) RJ production per cell cup in (mg) between both bee stocks. “***” represents statistically significant differences (Student’s *t*-test, p<0.05).

Similarly, RJ production per cell cup was significantly higher in Italian bee than Carniolan bee (t = 20.733, p = 0.001). Maximum RJ production per cell was higher in Italian bee colonies (238. 46 ± 1.96 mg), whereas 192.33 ± 1.06 mg per cell cup RJ was recorded for Carniolan bees.

### The effect of priming media on queen cell acceptance rate and RJ production

The effect of priming media on the queen cell acceptance rate and RJ production between Italian and Carniolan bee races are shown in Fig 3.

**Fig 3:** The effect of various priming media or coating material on queen cell acceptance rate (shows as mean ± SE) between Italian and Carniolan colonies. “^a, b, c, d, e^” different letter represents significant mean differences (Student’s *t*-test, p<0.05).

The queen cell acceptance rate significantly differed between Italian colonies with various priming material in plastic cell cups (F = 116.465, P = 0.001). Similarly, queen cell acceptance rate was significantly different within Carniolan bee colonies (F = 100.526, P = 0.001). In Italian bee colonies, the maximum queen cell acceptance rate was found in RJ primed plastic cup (81.16 ± 2.94%) compared to the other priming media. The percentage of less queen cell acceptance rate was (26.00 ± 1.15%) recorded for control group. In Carniolan bee colonies, the maximum queen cell acceptance rate was 61.67 ± 1.56% in RJ primed cups compared to control (19.33 ± 1.94%) (Table 1).

**Table 1:** The effect of various cup material priming media on the queen cell acceptance rate and royal jelly yield between Italian and Carniolan bee colonies.

Treatment	Italian bees	Carniolan bees	Italian bees	Carniolan bees	Italian bees	Carniolan bees
	Queen cell acceptance rate (%)		Weight (g) of royal jelly/ colony		Weight (mg) of royal jelly/ cell cup	
	Mean ± S. Error	Mean ± S. Error	Mean ± S. Error	Mean ± S. Error	Mean ± S. Error	Mean ± S. Error
Royal jelly	81.16 ± 2.94 a	61.67 ± 1.56 b	13.79 ± 0.52 a	11.29 ± 0.56 b	245.52 ± 3.67 a	197.07 ± 0.92 b
Diluted royal jelly	65.50 ± 2.47 a	53.17 ± 1.55 b	12.34 ± 0.54 a	10.18 ± 0.34 b	232.50 ± 2.56 a	189.40 ± 1.83 b
Honey solution	49.00 ± 1.71 a	43.50 ± 1.89 a	9.97 ± 0.62 a	9.30 ± 0.42 a	228.87 ± 4.07 a	182.10 ± 2.36 b
Sugar syrup	38.50 ± 1.18 a	31.83 ± 1.35 b	8.50 ± 0.63 a	7.50 ± 0.41 a	222.31 ± 2.96 a	175.26 ± 1.94 b
Control	26.00 ± 1.15 a	19.33 ± 1.94 b	7.13 ± 0.38 a	6.30 ± 0.37 a	208.80 ± 2.03 a	170.58 ± 2.07 b

In the row, the small different letter shows the significant difference between them (Student’s t-test, p<0.05).

The RJ production significantly differed in Italian bee colonies with various type of primed cups (F = 25.208, P = 0.001). In Italian bee colonies, the RJ production was 13.79 ± 0.52 g in case of coated cups with RJ and 12.34 ± 0.54 g in diluted RJ priming media (Fig 4A). The RJ production was 7.13 ± 0.38 g in control treatment. In Carniolan bees, mean weight (g) of RJ significantly differed by use of various priming media (F = 22.206, P = 0.001). The highest mean weight (11.29 ± 0.56 g) of RJ was recorded for RJ primed cups, whereas the lowest RJ production 6.30 ± 0.37 g was noted for control group (Fig 4A).

**Fig 4:** The effect of various priming media on royal jelly (mean ± SE) production of Italian and Carniolan colonies. (a) RJ production per colonies in grams after 72 hours of harvesting, (b) RJ production per cell cup in (mg) between both bee stocks. “^a, b, c^” different letter represents significant mean differences (Student’s *t*-test, p<0.05).

The mean weight of RJ per cell cup was statistically significant within Italian bee colonies with various primed cups (F = 18.427, P = 0.001). In Italian bee, the highest production per cell cup was 245.52 ± 3.67 mg with RJ priming, whereas the lowest RJ production (208.80 ± 2.03 mg/cell cup) was recorded for control treatment. The RJ production per cell cup significantly differed in Carniolan bee colonies with different primed cups (F = 31.695, P = 0.001). The highest weight of RJ per cell cup was 197.07 ± 0.92 mg was noted with RJ priming media, while the lowest RJ production per cell cup 170.58 ± 2.07 mg was observed for control treatment in Carniolan bee colonies (Fig 4B).

### The effect of different diets on queen cell acceptance and RJ production

The effect of various diets on queen cell acceptance rate and RJ production is described in Table 2. The queen cell acceptance rate significantly differed within Italian bee colonies fed with various diets (F = 129.575, P = 0.001). Similarly, queen cell acceptance rate was significantly different within the Carniolan bee colonies (F = 320.017, P = 0.001).

**Table 2:** The effect of various diets on the queen cell acceptance rate and royal jelly production between Italian and Carniolan bee colonies.

Treatment	Italian bees	Carniolan bees	Italian bees	Carniolan bees	Italian bees	Carniolan bees
	Queen cell acceptance rate (%)		Weight (g) of royal jelly/ colony		Weight (mg) of royal jelly/ cell cup	
Diet 1 = Pollen from a natural source	76.83±0.60 a	71.00± 1.53 b	14.06± 0.97 a	11.81± 0.31 b	243.42 ± 1.34 a	199.39± 1.70 b
Diet 2 = Pollen substitutes (soybean flour + brewer’s yeast powder)	67.17± 2.35 a	61.50± 1.38 a	12.50± 0.40 a	10.82± 0.23 b	231.52± 3.53 a	186.10± 2.41 b
Diet 3 = Sugar syrup (1:1 with water) only	37.83± 1.96 a	28.00± 0.73 b	8.86± 0.43 a	8.39± 0.40 a	219.95± 1.64 a	179.14± 1.67 b

In the row, the small different letter shows the significant difference between them (Student’s t-test, p<0.05).

There was no statistically significant difference for Carniolan bee colonies fed either on pollen or soybean flour plus brewer’s yeast powder (Fig 5).

**Fig 5:** The effect of various diets [Diet 1 = pollen from a natural source; Diet 2 = pollen substitutes (soybean flour + brewer’s yeast powder); Diet 3 = sugar syrup (1:1 with water)] on the queen cell acceptance rate (shows as mean ± SE) between Italian and Carniolan colonies. “^a, b, c^” different letter represents significant mean differences (Student’s *t*-test, p<0.05).

In respect to pollen diet, queen cell acceptance rate was significantly higher in Italian bee colonies than Carniolan bee colonies (t = 3.554, p = 0.005 (Table 2). In case of pollen substitutes (soybean flour plus brewer’s yeast powder), queen cell acceptance rate did not differ significantly between both races (t = 2.101, p = 0.062). Queen cell acceptance rate was 67.17 ± 2.35% in Italian bee colonies, whereas Carniolan bee colonies had 61.50 ± 1.38% acceptance rate (Table 2). In contrast, queen cell acceptance rate significantly differed between both bee races fed on sugar syrup (t = 4.709, p = 0.001) (Table 2). Queen cell acceptance rate was 37.83 ± 1.96% and 28.00 ± 0.73% in Italian and Carniolan bee races, respectively.

The effect of various diets on RJ production of Italian and Carniolan bee colonies is presented in Fig 6A and 6B. The RJ production significantly differed between Italian bee colonies fed on a various diet (F = 43.028, P = 0.001). In Italian bee colonies, RJ production was 14.06 ± 0.97 g with pollen diet and 12.50 ± 0.40 g with soybean plus yeast powder (Table 2). The RJ production was 8.86 ± 0.43 g in Italian colonies fed on sugar syrup. In Carniolan bees, the mean weight of RJ significantly differed with different diets (F = 29.468, P = 0.001). The RJ production did not differ significantly for the colonies fed on pollen (11.81 ± 0.31 g) or soybean flour plus brewer’s yeast powder (10.82 ± 0.23 g). The less RJ production 8.39 ± 0.40 g was noted in sugar syrup fed colonies (Fig 6A).

**Fig 6:** The effect of various diets [Diet 1 = pollen from a natural source; Diet 2 = pollen substitutes (soybean flour + brewer’s yeast powder); Diet 3 = sugar syrup (1:1 with water)] on royal jelly (mean ± SE) production in Italian and Carniolan colonies. (a) RJ production per colonies in grams after 72 hours of harvesting, (b) RJ production per cell cup in (mg) between both bee stocks. “^a, b, c^” different letter represents significant mean differences (Student’s *t*-test, p<0.05).

Similarly, the effect of various diets on RJ production per cell cup of Italian and Carniolan bee colonies is presented in Fig 6B. The mean weight of RJ per cell cup significantly differed between Italian bee colonies fed on various diet pollen, soybean flour plus brewer’s yeast powder and sugar syrup (F = 21.342, P = 0.001).

In Italian bee races, RJ production per cell cup was 243.42 ± 1.34 mg in pollen diet, 231.52 ± 3.53 mg in soybean plus yeast powder and 219.95 ± 1.64 mg in case of sugar syrup fed colonies. The RJ production per cell cup significantly differed in Carniolan bee colonies fed on various diets (F = 28.002, P = 0.001). In Carniolan bee colonies, mean weight of RJ per cell cup was 199.39 ± 1.70 mg in pollen diet, while 186.10± 2.41 mg in soybean flour plus brewer’s yeast powder diet and less RJ production per cell cup was 179.14 ± 1.67 mg was recorded for sugar syrup fed colonies (Table 2).

### The effect of seasons on queen cell acceptance and RJ production

The effect of season on queen cell acceptance rate and RJ production is given in Table 3. The queen cell acceptance did not differ significantly within Italian colonies during summer and winter seasons (t = 2.049, p = 0.057). The queen cell acceptance rate was 81.44 ± 1.09% in Italian bees during summer, whereas it was 77.44 ± 1.62% during winter (Fig 7A). In contrast, queen cell acceptance rate significantly differed within Carniolan bee colonies (t = 5.624, p = 0.001). In Carniolan bees, the queen cell acceptance rate was 66.44 ± 0.93% and 58.78 ± 0.97% during summer and winter seasons, respectively (Fig 7B).

**Fig 7:** The effect of various season on queen cell acceptance rate (shows as mean ± SE) between Italian and Carniolan colonies. “***” represents statistically significant differences (Student’s *t*-test, p<0.05).

**Table 3:** The percentage of queen cell acceptance rate and royal jelly yield between Italian and Carniolan bees during summer and winter seasons.

Season	Italian bees	Carniolan bees	Italian bees	Carniolan bees	Italian bees	Carniolan bees
	Queen cell acceptance rate (%)		Weight (g) of royal jelly/ colony		Weight (mg) of royal jelly/ cell cup	
Summer	81.44±1.09 a	66.44±0.93 b	13.83±0.39 a	10.74±0.24 b	242.57± 1.35 a	197.42± 2.70 b
Winter	77.44±1.62 a	58.78±0.97 b	12.04±0.19 a	9.29±0.31 b	225.98± 3.85 a	186.95± 2.61 b

In the row, the small different letter shows the significant difference between them (Student’s t-test, p<0.05).

The RJ production significantly differed between Italian bee colonies during summer and winter seasons (t = 4.152, p = 0.001). In Italian bee colonies, RJ production was 13.83 ± 0.39 g during summer and 12.04 ± 0.19 g in winter (Fig 8A). In Carniolan bees, the mean weight (g) of RJ significantly differed during summer and winter (t = 3.693, p = 0.002). The mean weight of RJ was 10.74 ± 0.24 g in summer season whereas it was 9.29 ± 0.31 g in the winter season (Fig 8A).

**Fig 8:** The mean weight of royal jelly (shows as mean ± SE) production between Italian and Carniolan colonies during summer and winter. (a) RJ production per colonies in grams after 72 hours of harvesting, (b) RJ production per cell cup in (mg) between both bee stocks. “^a, b, c^” different letter represents significant mean differences (Student’s *t*-test, p<0.05).

Similarly, the mean weight (mg) of RJ per cell cup significantly differed within Italian bee colonies during summer and winter (t = 4.061, p = 0.001). In Italian bees, the RJ production per cell cup was 242.57 ± 1.35 mg in summer, while it was 225.98 ± 3.85 mg during winter (Fig 8B). The RJ production per cell cup significantly differed within Carniolan bee colonies during both seasons (t = 2.788, p = 0.013). In Carniolan bee colonies, the maximum weight of RJ per cell cup was 197.42 ± 2.70 mg in summer, while 186.95 ± 2.61 mg in winter (**Fig 8B**).

## Discussion

This study identified queen cell acceptance rate and RJ production in Italian and Carniolan bee races. The average percentage of queen cell acceptance rate and RJ production was significantly higher in Italian race than Carniolan bee race.

Multiple factors may influence RJ production such genetics, inside population conditions, queen egg-laying capacity and environmental factors [6, 31, 36, 44, 45]. For instance, Hu [46] evaluated RJ production between high RJ-producing bees (RJBs) and Italian bees (ITBs). The results indicated that average RJ production in RJBs was 54.0 ± 3.4 g, while it was 3.7 ± 0.84 g in ITBs. Similarly, results supported that the average queen cell acceptance of RJBs (75%) was significantly higher than ITBs (10%). The RJBs could produce ≥10 kg RJ/year/ colony, confirming the feasibility of selection for this trait [29, 46]. The results were consistent with Hussain [45] who recorded that percentage of queen cell acceptance rate, RJ production per colony and cell cup was higher in Italian bee colonies than Carniolan bee colonies. In contrast, Şahinler and Kaftanoğlu [25] revealed that the average percentage of acceptance rate and production of RJ was higher in Carniolan followed by Mugla and Caucasian bees. However, in our experiment, RJ yield was lower than genetically modified bees in various part of the world.

Moreover, our results elucidated that cup cell priming media, diets and seasons significantly affected larval acceptance rate and RJ production of both bee races. The larval acceptance rate and RJ yield were higher in RJ-primed media than control in both bee races. Sharma [47] reported similar results, i.e., queen cell acceptance rate was higher in RJ-primed media followed by honey and sugar syrup. Furthermore, artificial sugar supplementation during RJ production is a common beekeeping practice, specifically in countries that have extremely hot and dry climates. However, bee-feeding with artificial supplements during RJ production remains a controversial subject. Unexpectedly our result did not determine the effect of various diet on RJ quality and its composition. Wytrychowski [48] reported that RJ quality such as physicochemical parameters (water, protein, amino acids, and 10-hydroxy-2-decenoic acid) remain consistent between the bee colonies feeding on soybean and yeast powder when compared with non-feeding RJ samples. Weiss [49] reported that stimulative feeding does not affect the queen acceptance rate and RJ production. In contrast, the botanical origin may affect the quantity, quality, and various components of RJ [38, 39]. The results of this study indicated that RJ production was significantly higher in summer seasons than winter seasons in both bee races. Hussain [45] revealed similar results that queen cell acceptance rate and RJ yield were higher in Italian bee hybrid than Carniolan bee hybrid during summer and winter seasons.

Generally, RJ production is affected by many intrinsic and external factors. It is necessary to investigate all possible methods that are applicable for any agro-ecological zones and other important factors to optimize RJ production using exploitation of genetic potential by breeding. In this regard, further studies are needed to determine the effect of various priming media, diets and seasons on RJ yield and quality parameters of Italian and Carniolan bee races.

## Conclusions

The results indicated that queen cell acceptance rate and RJ production was significantly higher in Italian bee race than Carniolan race. Different priming media significantly altered larval acceptance rate and RJ yield of both bee races. Furthermore, our result elucidated that the acceptance rate and RJ yield were affected by the various diets. The larval acceptance rate and RJ yield were significantly higher during summer than winter season. Further studies are needed to unveil the quality and components of RJ obtained from Italian and Carniolan bee races.
